# Comparative Analysis of Clinical Effects of the Cable-Pin System and Kirschner Wire Tension Band (TBW) Internal Fixation in the Treatment of the Olecranon Fracture

**DOI:** 10.1155/2022/3073121

**Published:** 2022-06-07

**Authors:** ChengZhi Rao, Hao Hu, RenYuan Tan

**Affiliations:** Department of Orthopedics, The First People's Hospital of Jiangxia, Wuhan City, Hubei Province 430200, China

## Abstract

**Objective:**

To explore the clinical effects of the cable-pin system and Kirschner wire tension band (TBW) internal fixation in the treatment of the olecranon fracture.

**Methods:**

Fifty patients with an olecranon fracture were treated in our hospital from April 2018 to March 2020. Patients were randomly divided into control and study groups. The control group was fixed with TBW, and the study group was fixed with the cable-pin system. The operation, the circumference difference between the injured limb and the healthy limb, the VAS score, the excellent and good rate, the recovery of the range of motion of the joint 1 year after operation, and the incidence of postoperative adverse reactions were compared between the two groups.

**Results:**

In terms of the operation of the two groups, the operation time, intraoperative blood loss, healing time, incision drainage, and hospital stay in the study group were lower than those in the control group (*P* < 0.05). In the comparison of the circumference difference between the injured limb and the healthy limb, there was no significant difference between the two groups before operation (*P* > 0.05), but the circumference difference between the injured limb and the healthy limb in the study group was lower than that in the control group at 24 hours, 72 hours, 7 days, and 30 days after operation, and the difference was statistically significant (*P* < 0.05). There was no significant difference in the VAS score between the two groups before operation, but 7-day VAS scores at 12 h, 24 h, and 72 h after operation in the study group were significantly lower than those in the control group (*P* < 0.05). The excellent and good rate in the study group was excellent in 18 cases, good in 5 cases, fair in 2 cases, excellent in 7 cases, good in 6 cases, fair in 8 cases, and poor in 4 cases in the control group, and the excellent and good rate in the study group (100.00%) was higher than that in the control group (84.00%), and the difference was statistically significant (*P* < 0.05). The patients in the two groups were followed-up for one year, and there were no shedding cases in the two groups. In terms of the recovery of range of motion one year after operation, the scores of elbow flexion, extension/degree, and elbow function in the study group were higher than those in the control group (*P* < 0.05), and the difference was statistically significant (*P* < 0.05). The incidence of postoperative adverse reactions in the study group (4.00%) was significantly lower than that in the control group (28.00%), and the difference was statistically significant (*P* < 0.05). The incidence of postoperative adverse reactions was significantly lower in the study group (4.00%) than that in the control group (28.00%), and the difference was statistically significant (*P* < 0.05), while only 1 patient in the study group had chronic pain, while 7 patients in the control group had incision ulcer (1 case), chronic pain (2 cases), and internal fixation loosening (4 cases). The difference was statistically significant (*P* < 0.05).

**Conclusion:**

The cable-pin system for the treatment of an olecranon fracture has the advantages of simple operation, fast fracture healing time, and low incidence of complications, which is a kind of orthopedic internal fixation consumable material in line with biomechanical requirements of the human body.

## 1. Introduction

Olecranon fractures are common intra-articular fractures, most common in adults, accounting for about 10% of perielbow fractures and 1% of systemic fractures [1]. In addition to small avulsion fractures, most fractures affect the articular surface of the semilunar notch, and the unevenness of the articular surface will cause limitation of the joint movement, delayed recovery, or traumatic arthritis, so accurate reduction and rigid fixation are effective measures to prevent the joint instability, prevent the occurrence of osteoarthritis, and restore the function of the elbow joint [2]. The treatment of such fractures can be divided into external fixation, manual reduction and external fixation, open reduction and internal fixation, and proximal resection [2]. Open reduction and internal fixation with Kirschner wire tension band is one of the commonly used methods for the treatment of this kind of fracture because of its firm fixation, simple operation, early functional exercise, and biomechanical characteristics of the elbow, but it has not solved the problems such as relatively large trauma of open reduction and internal fixation, serious injury of soft tissue peeling, and aesthetic influence of residual incision scar [3]. With the gradual improvement of patients' treatment requirements, it is an urgent problem to be solved in orthopedics and traumatology clinic to seek a treatment method with small incision, few complications, simple operation, safe, and effective.

With the continuous progress of orthopedic internal fixation devices, the cable-pin system is gradually applied in the fracture treatment in the comprehensive use of the principles of convergent tension band, tension nail, purse wrap, and convergent fixation [4]. The two ends of the system use a semithreaded cancellous bone compression screw and bone tunnel guide needle, respectively. The screw into the bone has a compression effect, and the steel cable is easy to tighten because of its flexibility, which can effectively prevent the screw from falling out [4]. Given that it combines the characteristics of biomechanical materials, after encircling, the cable has the dynamic compression effect of the tension band on the broken end of the patella fracture, forming the integration of the screw and cable, thus making the screw stronger and preventing the cable from further slipping [4]. The nail-cable interaction is greatly improved, and the cable can be adjusted according to the change of the fracture block and reduction mode during the operation, which makes it more flexible and efficient. It provides a stable biomechanical environment for fracture healing in the later stage [5]. Referring to relevant research reports at home and abroad [6–8], the orthopedic cable-pin system is mostly used in patellar fracture, total knee arthroplasty, and so on, but there are few reports on the ulnar olecranon fracture. In this study, we focused on the clinical effects of the cable-pin system and Kirschner wire tension band (TBW) in the treatment of the olecranon fracture.

## 2. Patients and Methods

### 2.1. Patient Information

Fifty patients with olecranon fracture were treated in our hospital from April 2018 to March 2020. In the control group, the age was 19–71 years old, with an average of (45.73 ± 2.64) years, including 13 males and 12 females, while in the study group, the age was 20–72 years old, with an average of (45.66 ± 2.56) years, including 11 males and 14 females. There was no statistical significance in the general data of the two groups. This study was approved by the Medical Ethics Association of our hospital. All patients signed an informed written consent.

The inclusion criteria were as follows: (1) closed, fresh, unilateral olecranon fracture with no combined injury; (2) no serious medical disease; and (3) orthopedic internal fixation consumables used in the operation were the cable-pin system or TBW.

The exclusion criteria were as follows: (1) patients with old and open fractures; (2) patients with ulnar coronal process fractures, radial head fractures, humeral intercondylar fractures, severe comminuted unstable fractures, and previous elbow joint dysfunction; (3) patients with severe organic diseases who cannot be tolerated by surgery; (4) patients under 18 years old or over 75 years old; and (5) pathological fractures.

### 2.2. Treatment Methods

Surgical methods: patients in both the groups were treated with posterior median incision of inferior 1/3 of the ulna on the affected side, simple fractures were treated with cloth towel forceps or point reduction forceps, and complex comminuted fractures could be temporarily fixed with 1-2 Kirschner wires. The cable-pin group: two Kirschner pins exceeding 5–6 cm of the fracture line were drilled longitudinally along the olecranon fracture, and cable-pin screws of 6.5 cm were screwed successively after tapping. It is noted that the thread should cross the fracture line, and the tail of the nail should be buried into the olecranon bone as far as possible, and then a channel perpendicular to the long axis of the ulna was drilled horizontally at about 6 cm at the distal end of the ulna and about 0.5 cm from the ulnar crest. After piercing the titanium cable from the horizontal channel, the titanium cable is wound and ligated with “8” after the ulnar olecranon, tightened, and locked with a binder. The TBW group: two Kirschner wires of 1.5–2.5 mm diameter were placed angularly through the proximal end of the olecranon fracture, and a transverse hole was drilled into a proper thickness steel wire at 1 point behind the ulnar ridge of 3–6 cm from the fracture line. The wire was fixed according to the “8” tension band principle. The tail of the Kirschner needle was reserved and bent, and the caudal end was placed into the bone cortex and pressed against the steel wire to prevent slippage. After the completion of effective fixation, patients in both groups were given passive elbow flexion with a range of 90–110 °to check the range of motion of the elbow joint, fracture reduction, and the firmness of the implant. After confirmation, the surgical incision was closed layer by layer.

The postoperative treatment: fluid replacement, prevention of infection, dehydration, and detumescence were routinely given after operation. On the first day after operation, patients were required to exercise passive flexion and extension of the elbow joint 2-3 times a day on the premise of strictly following the principle of “active, progressive, and enhanced” functional exercise. The active exercise of the elbow began 1 week after operation, and frequency was the same as before. The sutures were removed 2 weeks after operation and were reexamined 1, 2, 3, 6, and 12 months after operation. 24–48 weeks after operation, internal fixation was removed according to fracture healing of the patients.

### 2.3. Observation Index

#### 2.3.1. Operation Condition

The operation time, intraoperative blood loss, healing time, incision drainage, and length of hospital stay were calculated between the two groups. The clinical healing standard are as follows [9]: the fracture local shows no tenderness and longitudinal percussion pain; the fracture local shows no abnormal activity; X-ray shows that the fracture line is blurred and continuous callus passes through the fracture line. In the case of no external fixation, the upper limb can lift a weight of 1 kg for 1 minute; if there is no local deformation of the fracture for 2 weeks, then the first day of observation can be used as the clinical healing date of the fracture.

#### 2.3.2. Circumference Difference between Injured Limb and Healthy Limb

The measurement standard of the limb circumference difference between the injured limb and healthy limb. (1) Measuring tools: measuring with the same soft ruler to reduce measurement error. (2) Measurement method: the circumference of the most swollen part of the affected limb (the same part) was measured. (3) Measurement site: where the swelling of the injured limb is most obvious, take the same horizontal position on the healthy side and mark it for the next measurement. (4) Measurement time: the limb circumference was measured 1 hour before operation and 24 hours, 72 hours, 7 days, and 30 days after operation, and the average value was taken three times after operation.

#### 2.3.3. VAS Scoring

VAS scores of the two groups at 4 h, 8 h, 12 h, 24 h, and 48 h after operation were recorded [10]. With self-made 10 cm long VAS scale, the degree of pain increased from 0 (0: painless) to 10 (10: unbearable pain). The VAS scale is given to the patient, and let the patient give a clear score according to the number on the VAS scale according to the degree of pain and record the score value. If the patient has difficulty in reading or cannot understand the VAS ruler well, it can be explained to the patient, but not in place of the patient to give the score. If the patient is in unbearable pain, stop the experiment immediately, and give other effective ways of analgesia to relieve the patient's pain. The score criteria: 10—painless; 20 and 3—mild pain and bearable, respectively; 34–6—patient's pain and affect sleep, can bear; 47–10—patient has increasingly intense pain, unbearable pain, affect appetite, and affect sleep.

#### 2.3.4. Postoperative Excellent and Good Rate

Using the improved Cassebaum evaluation system [11]: (1) excellent: 15° elbow extension, 130° elbow flexion asymptomatic; (2) good: 30°elbow extension, 120° elbow flexion without symptoms; (3) 40° elbow extension, 90°–120° elbow flexion symptomatic; (4) poor: 40°elbow extension, elbow flexion <90°. Excellent and good rate = excellent rate + good rate + possibility rate.

#### 2.3.5. Recovery of Range of Motion of the Joint 1 Year after Operation

According to the comprehensive function score of the elbow joint (MEPS) [12]: excellent: more than 90 points; good: 75–89 points, medium: 60–74 points; poor: less than 60 points. During the follow-up of the patient for one year, the doctor scored the recovery of the elbow joint function of the affected limb and evaluated the improvement of the elbow joint function of the affected limb. At the same time, flexion, extension/degree of the elbow joint of the two groups were counted.

#### 2.3.6. Incidence of Postoperative Adverse Reactions

Incidence of adverse reactions: the incidence of incision ulcer, chronic pain, and internal fixation loosening were recorded in the two groups.

### 2.4. Statistical Analysis

Using SPSS21.0 statistical software, before statistical analysis, measurement data were tested by normal distribution and variance homogeneity analysis to meet the requirements of normal distribution or approximate normal distribution, expressed as $\bar{x}$ ± *s*, and repeated measurement data were analyzed by repeated measurement analysis of variance. The *T*-test was used to compare the two groups, *n* (%) was used to represent the counting data, and the *χ*^2^ test was used. The difference was statistically significant (*P* < 0.05).

## 3. Results

### 3.1. Comparison of Surgical Conditions

In terms of operation of the two groups, the operation time, intraoperative blood loss, healing time, incision drainage, and hospital stay in the study group were lower than those in the control group, and the difference was statistically significant (*P* < 0.05). All the results are shown in Table 1.

### 3.2. Comparison of Circumference Difference between Injured Limb and Healthy Limb

In comparison of the circumference difference between the injured limb and the healthy limb, there was no significant difference between the two groups before operation (*P* > 0.05), but the circumference difference between the injured limb and the healthy limb in the study group was lower than that in the control group at 24 hours, 72 hours, 7 days, and 30 days after operation, and the difference was statistically significant (*P* < 0.05). All the results are shown in Table 2.

### 3.3. Comparison of the VAS Score before and after Operation

There was no significant difference in the VAS score between the two groups before operation, but 7-day VAS scores at 12 h, 24 h, and 72 h after operation in the study group were significantly lower than those in the control group (*P* < 0.05), and the difference was statistically significant (*P* < 0.05). All the results are shown in Table 3.

### 3.4. Comparison of the Excellent and Good Rate after Operation

The excellent and good rate in the study group was excellent in 18 cases, good in 5 cases, fair in 2 cases, excellent in 7 cases, good in 6 cases, fair in 8 cases, and poor in 4 cases in the control group, and the excellent and good rate in the study group (100.00%) was higher than that in the control group (84.00%), and the difference was statistically significant (*P* < 0.05). See Table 4.

### 3.5. Comparison of the Recovery of the Joint Range of Motion One Year after Operation

Patients in the two groups were followed-up for one year, and there were no shedding cases in the two groups. Compared with the recovery of range of motion one year after operation, the scores of elbow flexion, extension/degree, and elbow function in the study group were higher than those in the control group, and the difference was statistically significant (*P* < 0.05). All the results are shown in Table 5.

### 3.6. Comparison of the Incidence of Postoperative Adverse Reactions

The incidence of postoperative adverse reactions in the study group was significantly lower than that in the control group (*P* < 0.05), and the difference was statistically significant (*P* < 0.05). The incidence of postoperative adverse reactions in the study group (4.00%) was significantly lower than that in the control group (28.00%), and the difference was statistically significant (*P* < 0.05). The incidence of postoperative adverse reactions was only 1 case in the study group and 7 cases in the control group (1 case), chronic pain (2 cases), and internal fixation loosening (4 cases), and the difference was statistically significant (*X*^2^ = 5.357, *P* < 0.05).

## 4. Discussion

The olecranon, which is located at the proximal end of the ulna, is a large curved process, which continuously forms the semilunar notch of the ulna with the coronal process in front of it. The concave part of the olecranon and the trochlear part of the humerus match together to form the humeral-ulnar joint. The sagittal position has the movement function of elbow flexion and extension, which is of great significance for maintaining the stability of the elbow [12]. In addition, since the ulnar olecranon is one of the important components of the elbow extension power device, the fracture in the olecranon also represents the fracture of the elbow extension device, and the patient often loses the function of active elbow extension [13]. The olecranon fracture is one of the common injuries of elbow, which is more common in adults, accounting for about 1.17% of systemic fractures [14]. With the continuous improvement of social material culture and living standards, the incidence of the olecranon fracture induced by a high energy compound injury is increasing year by year, except for a few olecranon tip avulsion fractures, most patients are intra-articular fractures involving the cartilage surface of the semilunar joint [13]. Owing to the interaction of extensor and flexor muscles of the elbow, the displacement of the fracture end is very prone to occur. If there is still a ladder on the articular surface after taking relevant treatment measures, it is very easy to result in many late complications [15]. At present, except for few minor fractures that can be treated conservatively, most fractures tend to be surgically treated, and different surgical treatment methods are available according to the characteristics and types of fractures [16]. For the treatment of intra-articular fractures, the AO technique has the following requirements: (a) anatomical reduction as far as possible; (b) stable fixation is given; (c) early functional activities; (d) paying attention to the protection of blood supply. The four aspects complement each other. Only after anatomical reduction of the end of the fracture can reliable and effective fixation be carried out. The protection of blood supply is conducive to fracture healing, and anatomical reduction and rigid fixation are precisely the premise of early joint activity and restoration of function. Therefore, in the treatment of the olecranon fracture with internal fixation, we should not only restore the original anatomical structure as much as possible but also pay attention to protect blood supply and soft tissue and also provide protection for early exercise [17]. Clinical practice has proved that good reduction, strong fixation, and early functional exercise can effectively avoid or reduce the occurrence of late complications.

In recent years, with the continuous development of the new internal fixation equipment and internal fixation technology, the main internal fixation methods for the treatment of the olecranon fracture include TBW internal fixation and ulnar olecranon locking compression plate internal fixation. These two methods are effective in the treatment of the olecranon fracture and how to select internal fixation methods and materials to treat the olecranon fracture properly, flexibly, and effectively [18] and rapidly promoting the recovery of patients' elbow function which is a very thorny problem in front of orthopedic surgeons [19]. The olecranon is an important mechanical fulcrum in the elbow extension device; once the injury causes the loss of active elbow extension function, the consequence is serious. At present, the clinical treatment for this disease tends to open reduction with internal fixation (ORIF). Under the premise of anatomical or functional reduction, ORIF can maintain solid and lasting fixation of the broken end of the olecranon fracture and reduce the occurrence of the olecranon semilunar articular surface unevenness and malunion after reduction [20]. TBW is the most commonly used method for the treatment of the olecranon fracture, but it also has some shortcomings. Some scholars have found that, in the process of postoperative functional exercise in patients with the olecranon fracture treated with TBW, the Kirschner needle is prone to complications, such as withdrawal of Kirschner wire, loosening, and subcutaneous irritation [21].

The cable-pin system is a new type of orthopedic internal fixation consumable material, which combines titanium cable and a semithreaded tension screw [22]. Although the mechanical properties of the cable-pin system and TBW are consistent with the basis and both are tension band principles, cable-pin system has the structural characteristics of the cancellous bone compression screw connected with a titanium cable and also has a binding device to prevent loosening of the system after operation. These characteristics can not only simplify the operation process of internal fixation of the olecranon fracture but also make the broken end of the olecranon fracture get long-term, firm fixation, and compression effect [22]. In accordance with the definition that promotes the repair and growth of the broken end of the fracture in stress direction, the loss of the fracture location after reduction can be avoided [23]. The experimental data show that due to its biological properties, the cable-pin system has no toxicity and rejection to implants from outside the human body and is harmless for a long time, owing to its more humanized design, flexible and portable operation, less stimulation to human tissue in the process of postoperative recovery, more convenient to take out, and less damage to body tissue. The cable-pin system has double advantages of the tension band and lag screw [24]. (1) Antirotation and compression: two semithreaded cancellous bone screws are inserted into the bone to fix and statically compress the broken end, which further avoids the possibility of the fracture and loosening in the process of rehabilitation exercise. (2) Reduction of complications: its biomaterials are nontoxic, the human body has no rejection to the implanted internal fixation, and it is less irritating to soft tissue, which avoids the possibility of complications, such as infection and skin nonunion. (3) The nailing cable is integrated, firm, and reliable and prevents the occurrence of the withdrawal of the nail and avoids the possibility of loosening the steel cable, and the two pull and press each other to make it more firm. (4) Flexible operation for comminuted patellar fracture, circular ligation is more beneficial to the knee joint functional exercise in the early stage. It is not only reflected in the intraoperative internal fixation, the operation is simple, but also reflected in the removal of internal fixation. In addition, in order to achieve a better therapeutic effect, attention should be paid to [25]: (1) the cable-pin system belongs to a fixation tool and not a reduction tool. After broken end reduction, the integrity of the articular surface is determined, and then the system is maintained and fixed. (2) The appropriate type of screw is selected, and the length should be determined according to the broken end, the fracture line, and the distance between the superior and inferior poles of the patella. Avoid being too long and too short to cause instability of the broken end of the patellar fracture, screw fracture, and loosening. (3) In addition, the grasp of the tightening force of the cable is in the hands of the operator. If the force is too high, the articular surface of the broken end of the patella will produce steps, and traumatic arthritis will occur. (4) When tightening the cable with a restrainer, make sure that the cable is completely tightened, and then locked. (5) When cutting the tail of the excess steel cable, it should be close to the edge of the binder to avoid excessively long stimulating soft tissue at the tail.

In terms of operation of the two groups, the operation time, intraoperative blood loss, healing time, incision drainage, and hospital stay in the study group were lower than those in the control group. In comparison of the circumference difference between the injured limb and the healthy limb, there was no significant difference between the two groups before operation, but the circumference difference between the injured limb and the healthy limb in the study group at 24 hours, 72 hours, 7 days, and 30 days after operation was lower than that, in the control group. VAS score comparison and preoperative comparison, there was no significant difference between the two groups; the study group postoperative 12 h, 24 h, and 72 h and the 7dVAS score was lower than the control group, the data difference was statistically significant. There are significant differences in the operative effect and the postoperative pain score between the two groups. It is considered that the cable-pin system integrates the principle of the AO tension band and the biomechanical characteristics of orthopedic materials, but it is more flexible, easy to fix, and remove. In addition, it has superior static strength, compared a with steel wire, and it has greater antifatigue strength, and because of its smaller design volume and less stimulation to soft tissue, the degree of postoperative pain is lower.

Combined with the results of this study, in terms of the postoperative excellent and good rate, the excellent and good rate of the study group (100%) was higher than that of the control group (84%), and the difference was statistically significant (*P* < 0.05). Patients in the two groups were followed-up for one year, and there were no shedding cases in the two groups. In terms of the recovery of range of motion one year after operation, scores of elbow flexion, extension/degree, and elbow function in the study group were higher than those in the control group, and the difference was statistically significant (*P* < 0.05). The incidence of postoperative adverse reactions in the study group (4.00%) was lower than that in the control group (28.00%), and the difference was statistically significant (*P* < 0.05). Analysis shows that, with the application of Kirschner wire tension band internal fixation, the muscle force of triceps brachii muscle is transformed into a limited, but changeable compression force between the broken ends of fractures, demonstrating that the greater the muscle strength, the greater the compressive stress between the broken ends of the fracture, so a kind of intermittent physiological stress beneficial to fracture healing is obtained, which is one of the clinical applications of the principle of elastic fixation [25]. However, this operation also has some shortcomings in practical application, such as the later Kirschner needle is easy to lose, return needle, and other shortcomings. Some patients also have pain and discomfort caused by local stimulation of the Kirschner needle or steel wire to the skin. In severe cases, it also has a certain impact on the functional exercise of the patients' elbows. The cable-pin system has the following advantages in the treatment of olecranon fracture [26]: (1) the binding device equipped with the cable-pin system can prevent the slippage and failure of the cable-pin system, which is beneficial to healing of the ulnar olecranon fracture with less subcutaneous irritation symptoms and fewer complications, such as wire loosening, fracture, and pintail slippage, and reduce the probability of secondary revision surgery. (2) The screw tail of the cable-pin system can be embedded in the bone cortex, which minimizes the pressure on the skin and soft tissue behind the olecranon of the elbow joint, and (3) the screw is connected with the titanium cable in the cable-pin system, which eliminates the need for reserved bending of the tail of the Kirschner needle during operation, and the operation is simple and firm.

## 5. Conclusion

In conclusion, the cable-pin system for the treatment of olecranon fracture has the advantages of simple operation, fast fracture healing time, and low incidence of complications. It is a kind of orthopedic internal fixation consumables in line with the biomechanical requirements of the human body. However, there are some shortcomings in this study, such as the short follow-up time and small sample size, which may offset the results of the study.

## Figures and Tables

**Table 1:** Comparison of surgical conditions between the two groups ($\bar{x}$ ± *s*).

Group	*N*	Intraoperative bleeding volume (ml)	Incision drainage (ml)	Healing time (d)	Operation time (min)	Length of stay in hospital (d)
C group	25	65.83 ± 4.52	20.48 ± 3.45	16.85 ± 3.31	89.83 ± 3.43	12.46 ± 3.11
R group	25	58.93 ± 2.35	15.96 ± 1.22	12.48 ± 1.22	74.85 ± 4.11	10.52 ± 3.35
*T*		6.772	6.175	6.193	13.991	2.122
*P*		0.001	0.001	0.001	0.001	0.039

**Table 2:** Comparison of the circumference difference between the injured limb and the healthy limb between the two groups before and after operation ($\bar{x}$ ± *s*, Points).

Group	*N*	Before operation	24 h after operation	72 h after operation	7 d after operation	30 d after operation
C group	25	1.94 ± 0.46	3.89 ± 0.64	2.38 ± 0.42	0.83 ± 0.33	0.55 ± 0.12
R group	25	1.93 ± 0.44	1.85 ± 0.35	1.38 ± 0.33	0.59 ± 0.21	0.21 ± 0.05
*t*		0.078	13.983	9.360	3.067	13.076
*P*		0.937	0.001	0.001	0.003	0.001

**Table 3:** Comparison of preoperative and postoperative VAS scores between the two groups ($\bar{x}$ ± *s*, points).

Group	*N*	Before operation	12 h after operation	24 h after operation	72 h after operation	7 d after operation
C group	25	4.59 ± 1.34	7.47 ± 1.25	6.59 ± 0.44	4.85 ± 0.52	2.84 ± 0.33
R group	25	4.58 ± 1.35	5.39 ± 1.35	3.58 ± 0.57	2.68 ± 0.63	1.38 ± 0.67
*t*		0.026	5.625	20.900	13.282	2.276
*P*		0.979	0.001	0.001	0.001	0.001

**Table 4:** Comparison of postoperative excellent and good rates between the two groups (*n*/%).

Group	*N*	Excellent	Good	But	Difference	Excellent and good rate
C group	25	7 (28.00)	6 (24.00)	8 (32.00)	4 (16.00)	84.00
R group	25	18 (72.00)	5 (20.00)	2 (8.00)	0	100.00
*χ* ^2^						4.347
*P*						0.037

**Table 5:** Comparison of the recovery of range of motion between the two groups one year after operation ($\bar{x}$ ± *s*).

Group	*N*	Elbow flexion (degree)	Elbow extension (degree)	Elbow function score
C group	25	106.83 ± 6.93	7.83 ± 1.36	65.89 ± 4.11
R group	25	128.68 ± 2.55	13.74 ± 2.35	78.92 ± 3.66
*χ* ^2^		14.749	10.883	11.838
*P*		0.001	0.001	0.001

## Data Availability

The datasets used and analyzed during the current study are available from the corresponding author upon reasonable request.
